The article "Melatonin attenuates the TLR4-mediated inflammatory response through MyD88- and TRIF-dependent signaling pathways in an in vivo model of ovarian cancer" was retracted in 2025. Reasons: duplicated images; overlap with earlier publications; unreliable data; concerns about the images.

# Melatonin attenuates the TLR4-mediated inflammatory response through MyD88- and TRIF-dependent signaling pathways in an in vivo model of ovarian cancer

**DOI:** 10.1186/s12885-015-1032-4

**Published:** 2015-02-06

**Authors:** Luiz Gustavo A Chuffa, Beatriz A Fioruci-Fontanelli, Leonardo O Mendes, Fábio R Ferreira Seiva, Marcelo Martinez, Wagner J Fávaro, Raquel F Domeniconi, Patrícia FF Pinheiro, Lucilene Delazari dos Santos, Francisco Eduardo Martinez

**Affiliations:** 1 Department of Anatomy, Institute of Biosciences, UNESP – Universidade Estadual Paulista, Botucatu, SP Brazil; 2 Institute of Biology, State University of North of Parana, UENP - Campus Luiz Meneghel, Bandeirantes, PR Brazil; 3 Department of Morphology and Pathology, UFSCar – Universidade Federal de São Carlos, São Carlos, SP Brazil; 4 Department of Anatomy, Cell Biology and Physiology and Biophysics, UNICAMP – Universidade de Campinas, Campinas, SP Brazil; 5 Center for the Study of Venoms and Venomous Animals (CEVAP), UNESP - Univ Estadual Paulista, Botucatu, SP Brazil

**Keywords:** Ovarian cancer, Melatonin, Inflammation, TLR4, MyD88, TRIF

## Abstract

**Background:**

Toll-like receptors (TLRs) are effector molecules expressed on the surface of ovarian cancer (OC) cells, but the functions of the TLR2/TLR4 signaling pathways in these cells remain unclear. Melatonin (mel) acts as an anti-inflammatory factor and has been reported to modulate TLRs in some aggressive tumor cell types. Therefore, we investigated OC and the effect of long-term mel therapy on the signaling pathways mediated by TLR2 and TLR4 via myeloid differentiation factor 88 (MyD88) and toll-like receptor-associated activator of interferon (TRIF) in an ethanol-preferring rat model.

**Methods:**

To induce OC, the left ovary of animals either consuming 10% (v/v) ethanol or not was injected directly under the bursa with a single dose of 100 μg of 7,12-dimethylbenz(a)anthracene (DMBA) dissolved in 10 μL of sesame oil. The right ovaries were used as sham-surgery controls. After developing OC, half of the animals received i.p. injections of mel (200 μg/100 g b.w./day) for 60 days.

**Results:**

Although mel therapy was unable to reduce TLR2 levels, it was able to suppress the OC-associated increase in the levels of the following proteins: TLR4, MyD88, nuclear factor kappa B (NFkB p65), inhibitor of NFkB alpha (IkBα), IkB kinase alpha (IKK-α), TNF receptor-associated factor 6 (TRAF6), TRIF, interferon regulatory factor 3 (IRF3), interferon β (IFN-β), tumor necrosis factor alpha (TNF-α), and interleukin (IL)-6. In addition, mel significantly attenuated the expression of IkBα, NFkB p65, TRIF and IRF-3, which are involved in TLR4-mediated signaling in OC during ethanol intake.

**Conclusion:**

Collectively, our results suggest that mel attenuates the TLR4-induced MyD88- and TRIF-dependent signaling pathways in ethanol-preferring rats with OC.

## Background

Ovarian cancer (OC), which affects approximately 1 in 70 women, is among the most lethal gynecological malignancies and exhibits a poor prognosis when diagnosed during the late stage (<50% with a 5-year survival rate) [1]. Unfortunately, early-stage OC presents with no apparent symptoms, and no effective screening tool is currently available [2]. OC has been presumed to arise from lesions involving the ovarian surface epithelium (OSE) or ovarian epithelial inclusion cysts [1,2], which exhibit morphological characteristics of the reproductive tract epithelium (or Mullerian duct). Resistance to chemotherapy is the primary factor that hinders the long-term treatment of OC [2], and paclitaxel resistance has been recognized to induce recurrent OC and protumor activities [3].

TLRs are cell surface sensors that can initiate pathways to stimulate cell proliferation and chemoresistance, as well as recruiting immune cells to provide support for cancer progression [4]. It has been documented that TLR4 plays important roles in promoting the immune escape of several human cancer cells, including OC cells [5,6]. Furthermore, TLR4-mediated signaling is associated with the metastatic potential of tumor cells [7]. TLRs generally signal via a MyD88-dependent pathway, leading to a proinflammatory response. MyD88-mediated signaling promotes the early activation of NFkB, a nuclear factor that is responsible for the production of many proinflammatory cytokines, such as interleukin (IL)-6, IL-8, and TNF-α and is related to the immune response, cell adhesion, proliferation, angiogenesis, and apoptosis [8,9]. Conversely, a MyD88-independent pathway involves TRAM and, instead of MyD88, stimulates TRIF signaling, leading to late-phase activation of NFkB and induction of IRF3, which increases the production of IFN and IFN-inducible gene products [10].

Because ethanol (EtOH) intake produces a variety of co-carcinogenic and pro-inflammatory effects and seems to positively regulate TLR2/TLR4, IkBα, NFkB, and TNF-α [11], the combination of induced OC and EtOH intake results in the appropriate histological and molecular patterns that are needed to evaluate new chemotherapeutic compounds. Thus, we have previously proposed a useful, ethanol-preferring rat model for studying OC, and, notably, long-term mel therapy significantly reduced OC masses and the incidence of adenocarcinomas [12]. EtOH consumption by these animals is associated with cumulative incidence of serous papillary carcinoma and upregulation of Her-2-signaling pathway by OC cells [13].

Mel (*N*-acetyl-5-methoxytryptamine) is an indoleamine produced by the pineal gland, with maximal secretion at night [14]. The nighttime surge of mel has been suggested to serve as a "natural restraint" for tumor initiation, promotion, and progression [15]. Mel has been indisputably implicated as a therapeutic agent, including in the treatment of reproductive cancers [16,17]. Due to its versatility, mel has been recognized as having antioxidant, oncostatic, and immunomodulatory properties [18,19]. Numerous reports have shown that mel modulates early and late NFkB signaling during inflammation [20,21], thus resulting in changes in the expression of genes such as IL-1, IL-6, IL-12, and TNF-α [22]. Furthermore, some cytokines (IL-2, IL-6, and IL-12) and factors (TNF-α and IFNs) displaying immunotherapeutic potential have been associated with mel and are under investigation as adjuvant therapies for cancer [23,24]. Notably, the administration of mel significantly suppresses the expression of TLR4 and, in turn, MyD88, cytosolic IkBα, and nuclear NFkB p65 after ischemia/reperfusion in rats. Taken together, the reduction of p38 MAPK, NFkB, TNF-α, and IL-6 expression occurs due to an indirect decrease in the MyD88 protein levels [25]. Despite considerable efforts to understand the activation of the TLR2 and TLR4 signaling pathways, the exact mechanism(s) by which mel acts in the OC microenvironment remain unclear.

To better understand this issue, the present study was designed to investigate OC and the effect of long-term mel therapy on the signaling pathways mediated by TLR2 and TLR4 via MyD88 and TRIF in an ethanol-preferring rat model.

## Methods

### Animals and experimental design

Eighty 60-day-old adult UChB (a model of ethanol-preferring rats that was developed by selective breeding) female rats weighing 200–230 g were obtained from the Department of Anatomy, Bioscience Institute/Campus of Botucatu, Univ Estadual Paulista (UNESP). The rats were individually housed in polypropylene cages containing laboratory-grade pine shavings as bedding and were maintained under constant room temperature (RT; 23 ± 1°C) and lighting conditions (12-h light/dark cycle, with the lights switched on at 6 a.m.). Filtered tap water and standard rodent chow (3074 SIF, Purina Ltda., Campinas, SP, Brazil) containing (by weight) 19.90% protein, 30.03% carbohydrate, 3.80% fat, and 13.36% fiber, representing 3.00 kcal/g metabolizable energy, were provided *ad libitum*. All animals were divided into two arms (n = 40/group): the EtOH group, in which the rats were provided with access to a 10% (v/v) ethanol solution *ad libitum* (free choice of water or ethanol), and a control group, which was composed of ethanol-naïve rats without access to ethanol. When the ethanol-preferring rats reached 65 days of age, they were given a choice between two bottles containing either water or a 10% (v/v) ethanol solution *ad libitum* for 15 days. The animals displaying EtOH consumption greater than 2.0 g EtOH/kg/day (ranging from 4 to 5 g EtOH/kg/day) were selected according to the procedure described by Chuffa et al. [26,27]. In this study, the preference rate associated with ethanol-seeking behavior was approximately 70%.

After OC development (260-days-old), the animals (n = 40) designated to receive mel (M-5250, Sigma-Aldrich, St. Louis, MO, USA) were administered i.p. doses of 200 μg/100 g b.w. dissolved in 0.04 mL of 95% EtOH and then diluted in 0.3 mL of 0.9% NaCl (vehicle) to a final concentration of 0.3 mg/mL. The daily injections were administered nocturnally (between 18:30 and 19:00, Zeitgeber time (ZT) 13, Figure 1B) for 60 consecutive days (Figure 1A) [28,29].

**Figure 1:** **Experimental design, OC development, and mel treatment. (A)** Timeline for EtOH intake selection, ovarian tumor induction, and mel therapy (days). **(B)** Basic protocol used for daily melatonin administration based on ZT and corresponding to the environmental circadian time. ZT 13: time point of melatonin administration; ZT 22: time point of euthanasia. **(C)** Cumulative incidence (%) of OC from 120 to 260 days of age in animals receiving EtOH or EtOH + DMBA. **(D)** Macroscopic and histopathological characteristics of the OC tissue in the ethanol-drinking animals. Mel therapy efficiently reduced the tumor size but exerted no effect on tissue morphology (tumor = left ovary, bar = 20 μm; sham = right ovary, bar = 50 μm). **(E)** The plasma mel levels (pg/mL) prior to treatment initiation (day 0) and after 30 and 60 days of treatment. **(F)** The tumor volume (mm^3^) was recorded throughout the treatments. ^a^P < 0.05 vs. Group OC; ^b^P < 0.05 vs. Group OC + EtOH.

Finally, the rats were divided into four groups (n = 20): Group OC, composed of DMBA-induced animals that did not consume EtOH; Group OC + EtOH, composed of DMBA-induced animals that consumed 10% (v/v) EtOH during ovarian tumor development (OTD); Group OC + Mel, composed of DMBA-induced animals that received mel as a therapy; and Group OC + EtOH + Mel, composed of DMBA-induced animals that consumed 10% (v/v) EtOH during OTD and received mel as a therapy. After these procedures, the females were anesthetized and euthanized by decapitation (during the early morning at 4 a.m. or at ZT 22, which corresponded to the environmental circadian time; Figure 1B) for sample collection.

### Ethical statement

The use of laboratory animals in this study was approved by the Ethical Committee of the Institute of Bioscience/UNESP (CEEA – Permit Number: 382). The guide for the care and use of laboratory animals, published by National Academy of Science, was strictly followed in all experiments. To minimize pain, suffering or distress during experimentation, all of the animals were anesthetized with ketamine (50 mg/kg) and xylazine (10 mg/kg) prior to decapitation so that they were rendered unconscious.

### Ovarian tumor induction procedure

After selection based on ethanol consumption, all of the animals (n = 80) were anesthetized using 10% ketamine (60 mg/kg, i.p.) and 2% xylazine (5 mg/kg, i.p.) during the estrous phase, and the left flank region of the skin was cleaned with iodine and 70% EtOH. A 2-cm incision through the skin and the abdominal muscles was performed, and the ovaries were accessed after grasping the fat pad near the left kidney. The left ovary was injected directly under the bursa with a single dose of 100 μg of DMBA (Sigma Chemical Co, St Louis, MO) dissolved in 10 μL of sesame oil, which was used as the vehicle [30], and was returned intact to the body cavity. The muscle and skin layers were closed using a 3–0 silk suture (Ethicon, Inc., Juarez, MX). Sham surgery was conducted on the right ovary by administering only the vehicle. An antibiotic (10^5^ units of benzylpenicillin potassium) was administered i.p. for prophylactic treatment. Over the next 180 days, the rats were monitored, and tumor development was observed via ultrasonography. The ovary size (volume and diameter) was used as a comparative parameter during OC development, and high-grade serous papillary carcinomas were subjected to treatment.

### Determination of plasma mel concentrations

After blood collection (4 a.m.), mel was extracted from plasma (n = 20 samples/group) using HPLC-grade methanol and was separated on HPLC column (Sep-Pak Vac C-18, reverse phase, 12.5 nm; Water Corporation, Milford, MA, USA). Thereafter, 50 μL of the reconstituted samples were assayed using a Coat-a-count Melatonin ELISA Kit and were immediately read at 405 nm. The intra-assay coefficient of variation was 4%, and all of the samples were assayed in duplicate to avoid inter-assay variability. All of the reagents and microtiter plates were provided by IBL International (Hamburg, Germany). The concentrations of mel are presented as pg/mL.

### Immunohistochemistry

For immunohistochemistry, sections of OC tissue (n = 10/group) were deparaffinized in xylene based on the areas previously identified during the morphological characterization. Thereafter, tissue sections were microwaved (700–800 W) while immersed in 0.01 M sodium citrate buffer, pH 6.0, for 3 × 5 min for antigen retrieval. After blocking endogenous peroxidase activity with 3% hydrogen peroxide and 97% methanol, the tissues were incubated in 3% bovine serum albumin (BSA) for 1 h to eliminate non-specific binding. Subsequently, OC tissue sections were incubated in a humidified chamber overnight at 4°C with primary antibodies (Abcam, Cambridge, UK): rabbit polyclonal anti-TLR2 (1:100), mouse monoclonal anti-TLR4 (1:100), rabbit polyclonal anti-MyD88 (4 μg/ml), rabbit polyclonal anti-IkBα (1:50), rabbit monoclonal anti-IKKα (1:50), rabbit polyclonal anti-NFkB p65 (1:100), rabbit monoclonal anti-TRAF6 (1:50), rabbit polyclonal anti-TRIF (1:100), and rabbit monoclonal anti-IRF3 (1:100). After immunoreaction, the slides were washed in TBS-T buffer and incubated with secondary antibody (Polymer Anti-Mouse IgG or Anti-Rabbit - DAKO ® CYT) at RT for 1 h. Then, the slides were reacted with chromogen diaminobenzidine (DAB; Sigma, St. Louis, MO, USA) for 5 min. Finally, tissue sections were counterstained with hematoxylin. Negative controls were generated by omitting the primary antibody. The IHC results were analyzed by two pathologists under a Zeiss Axiophot II microscope (Carl Zeiss, Oberkochen, Germany) based on the levels of staining intensity, which were scored as absent (0), weak (+), moderate (++), or strong (+++) immunoreactivity.

### Immunofluorescence assays

Epithelial OC cells were cultured, washed with phosphate-buffered saline (PBS; sodium chloride, potassium chloride, dihydrogen phosphate, and disodium hydrogen phosphate), fixed in 4% paraformaldehyde for 10 min, and permeabilized with PBS at RT. Nonspecific binding sites were blocked with 1% BSA for 60 min. The samples were incubated with the anti-NFkB p65 primary rabbit polyclonal antibody (dilution 1:100, ab7970, Abcam, Cambridge, MA, USA) overnight at 4°C, followed by a secondary polyclonal anti-rabbit IgG conjugated to FITC (1:200, sc-2012, Santa Cruz Biotechnology, Inc., Santa Cruz, CA, USA) for 1 h at RT. Nuclei were stained with 6-diamidino-2-phenylindole (DAPI, 5 min) at RT. Primary and secondary antibodies were diluted in blocking buffer (1% BSA). For negative immunolabeling, no primary antibody was added. The immunopositive cells were analyzed using a fluorescence microscope (Zeiss Axiophot II, Oberkochen, Germany) at 40× magnification (immunofluorescence: excitation 590 nm, emission filter 650 nm) and for DAPI staining (excitation 365 nm, emission filter 435–485 nm). The quantification of relative fluorescence in the merged images was performed using Image J software.

### Immunoblotting and protein quantification

After mel therapy, the abdominal cavity was opened, the OC samples were rapidly removed, and 100-mg tissue samples were frozen in liquid nitrogen and stored at −80°C. The tissues were microdissected (only areas containing serous papillary tumors were obtained from the ovaries) and homogenized using 10× RIPA lysis buffer (Pierce Biotechnology, Rockford, IL, USA) supplemented with a cocktail of protease inhibitors (Sigma Chemical Co.). Aliquots of 1:10 (v/v) dilutions of Triton X-100 were added to the homogenates, and samples were placed on dry ice with agitation for 2 h to improve extraction. The lysates were centrifuged at 21,912 g for 20 min at 4°C to remove insoluble material, and total protein was measured through colorimetric determination. All protein samples were dissolved in 1.5X Laemmli buffer and used for SDS-PAGE (Bio-Rad Laboratories, Hercules, CA, USA). The same amount of protein (70 μg) was loaded per well and resolved on preformed 4-12% acrylamide gradient gels (Amersham Biosciences, Uppsala, Sweden) using a Tris-glycine running buffer electrophoresis system (60 mA for 2 h). After electrophoresis, total protein samples were electro-transferred (200 mA for 1.5 h) to nitrocellulose membranes in Tris-glycine-methanol buffer. Kaleidoscope Prestained Standards (Bio-Rad, Hercules, CA, USA) were used as molecular weight markers. Thereafter, the membranes were blocked with TBS-T solution containing 3% BSA at RT for 60 min and then incubated at 4°C overnight with the following antibodies (1:500 in 1% BSA): TLR2, TLR4, MyD88, IkBα, IKK-α, NFkB p65, NFkB p50, TRAF6, TRIF, and IRF-3 (Abcam, Cambridge, UK). This treatment was followed by 3 × 5 min washes in TBS-T solution and incubation for 2 h at RT with rabbit or mouse HRP-conjugated secondary antibodies (diluted 1:1000 in 1% BSA; Sigma-Aldrich Chemicals, St. Louis, MO, USA). After sequential washes in TBS-T, the signals were developed using an ECL detection kit (Thermo Scientific). Immunoreactive bands were obtained from individual blots of 10 rats/group using image analysis software (NIS-Elements, Advanced Research, Nikon). β-actin (cytosolic extract) and Lamin B1 (nuclear extract) were used as endogenous positive controls, and the results were expressed as the means ± SD. The protein concentrations are presented as the percentage of the optical density (band intensity-background) relative to the positive control.

### Subcellular fractionation

Cytosolic and nuclear extracts were obtained from OC cells using NE-PER nuclear and cytoplasmic extraction reagents (Thermo Scientific, Rockford, IL) according to the manufacturer's instructions. Equivalent amounts of the cytoplasmic and nuclear fractions were boiled in SDS lysis buffer for Western blot analysis. To ensure no cross-contamination occurred, specific biomarkers for the cytosolic and nuclear fractions were used.

### Elisa assays

The concentrations of IFN-β (cat. R1F00), TNF-α (cat. RTA00), IL-6 (cat. R6000B), and IL-8 (cat. D8000C) were measured using equal amounts of the supernatants of the OC samples. Commercial coated-a-coat rat ELISA kits were provided by R&D Systems (Minneapolis, MN, USA).

### Statistical analysis

The values are presented as the means ± standard deviation (SD), and data analyses were performed using two-way analysis of variance (ANOVA) for two independent factors (EtOH consumption and mel treatment). Significant results were subjected to *post-hoc* analysis using Tukey's test, and significance was set at P < 0.05. GraphPad Instat Version 4 statistical software and *Sigma Plot Version 12.5* graphing software were used.

## Results

### OC development and mel therapy

Although the cumulative OC incidence was slightly increased after the combination of DMBA with EtOH intake (Figure 1C), no apparent difference in the OC phenotype was observed following EtOH consumption. To confirm the effect of mel on this rat model of OC, macroscopic and microscopic analyses were frequently performed (Figure 1D); although mel therapy reduced the size of the OC, their serous papillary aspects with markedly pleomorphic nuclei were unchanged after mel treatment (Figure 1D). Notably, we measured the plasma mel levels to validate its concentration during long-term therapy in animals consuming or not consuming EtOH and exhibiting OC. As expected, a high concentration of mel was found in both the OC + Mel and OC + EtOH + Mel groups after 30- and 60-day treatment (Figure 1E). As a consequence of mel treatment, the tumor volume was reduced after 30 days (by about 29% and 34.8% for the OC and OC + EtOH groups, respectively; Figure 1F) and 60 days (by about 48% and 54.2% for the OC and OC + EtOH groups, respectively; Figure 1F).

### Mel differentially regulated the expression of TLR2, TLR4, and MyD88 in OC of EtOH-preferring rats

In response to mel treatment, TLR2 expression and immunostaining were increased (1.22-fold increase vs. OC) in the epithelium of serous papillary carcinoma (Table 1, Figure 2A, B, M, N). However, the combination of EtOH with mel caused a significant downregulation of TLR2 (1.54- and 1.16-fold reduction vs. OC + Mel and OC + EtOH, respectively, Table 1, Figure 2B-D, M, N). In contrast, mel therapy negatively regulated TLR4 (1.23-fold reduction vs. OC; Table 1, Figure 2E, F, M, O) and MyD88 (1.30-fold reduction vs. OC; Table 1, Figure 2I, J, M, P) in these cells. The effects of mel therapy and/or EtOH intake on the TLR2- and TLR4-induced MyD88-mediated signaling pathways are presented in Figure 2Q.

**Table 1:** **Scoring of immunohistochemical staining of OC cells**

	Treatments			
	OC	OC + Mel	OC + EtOH	OC + EtOH + Mel
TLR2	+	++	+	0
TLR4	+++	+	+++	++
MyD88	++	0	++	+
IKK-α	+	0	++	++
IkBα	++/+++	0/+	++/+++	0/+
NFkB p65	+++	0/+	+++	++
TRAF6	++	+	+	+
TRIF	+/++	+	+/++	+
IRF3	+++	++	+++	++/+++

OC staining were interpreted by pathologist visual scoring as 0 (no staining), + (<10% of carcinoma staining), ++ (10-50% of carcinoma staining), or +++ (>50% of carcinoma staining). N = 10 animals/group. Five selected OC sections were analyzed per animal.

**Figure 2:** **Immunohistochemical localization and Western blot analysis of TLR2, TLR4 and MyD88 in serous papillary ovarian carcinoma.** The immunoreactivity for TLR2 was moderate in the surface epithelium of OC + Mel **(B)** compared to OC animals **(A)** (arrows). Weak immunoreactivity for TLR2 was found in OC + EtOH animals **(C)** but was more pronounced in OC + EtOH + Mel animals **(D)**. TLR4 immunoreactivity was intense in the surface epithelium, but not in the stroma, of the OC **(E)** and OC + EtOH groups **(G)** (arrows). Weak immunoreactivity for TLR4 was observed in the OC + Mel group **(F)** (arrow), and moderate TLR4 reaction was detected in the epithelium of the OC + EtOH + Mel group **(H)** (arrow). Moderate MyD88 reaction was observed in the epithelium of the OC group **(I)** (arrow), in contrast to very weak immunoreactivity for MyD88 in the OC + Mel group **(J)** (arrow). The OC + EtOH **(K)** and OC + EtOH + Mel groups **(L)** displayed moderate and weak signals for MyD88, respectively (arrows). Bar = 20 μm. Negative controls were used. **(M)** Representative TLR2, TLR4, and MyD88 expression profiles in extracts (70 μg protein) pooled from 10 samples/group (upper panel). **(N–P)** Extracts obtained from individual rats were used for densitometric analysis of the TLR2, TLR4, and MyD88 levels following normalization to the β-actin. All results are expressed as the means ± SD (n = 10 animals/group). ^a^P < 0.05 vs. OC; ^b^P < 0.05 vs. OC + Mel and ^c^P < 0.05 vs. OC + EtOH. **(Q)** Schematic representation of the TLR2 and TLR4 signaling pathways via MyD88 and IRAK intracellular cascade, leading to NFkB activation, in a typical ovarian carcinoma cell. TLR2 is upregulated by mel and downregulated by EtOH + Mel, whereas TLR4 is downregulated by mel. Mel therapy also negatively regulates MyD88 expression. mel: melatonin; EtOH: ethanol; IRAK: IL-1 receptor-associated kinase; TRAF6: TNF receptor-associated factor 6; TAK1: TGF-B-activated kinase 1; NFkB: nuclear factor kappa B.

### The downregulation of NFkB signaling is enhanced by Mel regardless of EtOH intake

The involvement of the NFkB pathway during mel or EtOH treatment was determined in cytosolic and nuclear extracts of OC cells by analyzing the expression of IKK-α, IkBα, and NFkB p65/p50. Notably, IKK-α and IkBα were downregulated by mel therapy (1.25- and 1.37-fold reduction vs. OC; Table 1, Figure 3A, B, E, F and Figure 4A-C). In contrast, IKK-α was upregulated after EtOH intake or EtOH + Mel treatment (1.15- and 1.35-fold vs. OC and OC + Mel, respectively; Table 1, Figure 3C, D and Figure 4A, B). The combination of mel with EtOH reduced IkBα expression (1.42-fold decrease vs. OC + EtOH; Table 1, Figure 3G, H and Figure 4A, C), similar to mel treatment alone. As expected, the epithelial OC cells were NFkB p65-positive in the cytoplasm and nucleus (Table 1, Figure 3I) and became strongly immunopositive after EtOH intake (Table 1, Figure 3K). Surprisingly, mel alone induced the downregulation of cytosolic NFkB p65 and p50 (0.2- and 0.25-fold reduction, respectively, vs. OC; Figure 4A, D, E) and nuclear NFkB p65 (0.18-fold reduction vs. OC; Figure 4A, F, G); presumably, a negligible amount of the NFkB p65/p50 complex was translocated as a dimer to the nucleus. In addition, mel satisfactorily downregulated NFkB p65 in animals with OC that consumed EtOH (Figure 3L and Figure 4A, D, F, G). Briefly, Figure 4H shows the positive or negative regulatory effects of mel or EtOH on NFkB activation in the OC cells "in vivo". Immunofluorescence assays revealed the expression level and localization of cytosolic/nuclear NFkB p65 in OC cells. Mel therapy efficiently resulted in downregulation of NFkB p65 expression (Figure 4I, J; level of fluorescence reduced from 97% ± 10.2 (OC) to 66% ± 14.6 (OC + Mel)). In contrast, the levels of nuclear and cytosolic NFkB p65 were significantly increased by EtOH intake and were drastically decreased after mel treatment (Figure 4K, L; level of fluorescence 168% ± 19.2 (OC + EtOH) vs. 84% ± 11.6 (OC + EtOH + Mel)).

**Figure 3:** **Immunohistochemical localization of IKK-α, IkBα, and NFkB in serous papillary ovarian carcinoma.** Immunoreactivity for IKK-α was weak in the OC group **(A)** and absent from the OC + Mel group **(B)**. Moderate reaction for IKK-α was detected in the OC + EtOH **(C)** and OC + EtOH + Mel animals **(D)**. Immunoreactivity for IkBα was moderate to high in the surface epithelium of the OC **(E)** and OC + EtOH groups **(G)** and was weak in the OC + Mel **(F)** and OC + EtOH + Mel groups **(H)**. Strong immunoreactivity for NFkB was detected in the epithelium of the pappilae of the OC **(I)** and OC + EtOH groups **(K)**. The OC + Mel **(J)** and OC + EtOH + Mel groups **(L)** displayed weak and moderate signals for NFkB, respectively (arrows; Bar = 20 μm).

**Figure 4:** **Western blot analysis of IKK-α, IkBα, and NFkB in serous papillary ovarian carcinoma.** Representative protein profiles **(A)** of cytosolic and nuclear extracts (70 μg protein) pooled from 10 samples/group. **(B–G)**. Extracts obtained from individual rats were used for densitometric analysis of the protein levels following normalization to β-actin or LaminB1. The results are expressed as the means ± SD (n = 10 animals/group). ^a^P < 0.05 vs. OC; ^b^P < 0.05 vs. OC + Mel; and ^c^P < 0.05 vs. OC + EtOH. **(H)** The canonical pathway that leads to the activation of NFkB after a ligand binds to its specific receptor. Internal signaling results in the phosphorylation of IkBα by the IKK complex, leading to the ubiquitylation and degradation of NFkB via proteasome. The NFkB p65/p50 complex translocates to the nucleus to initiate the transactivation of target genes related to the inflammatory process. Mel induces the downregulation of IKK-α, IkBα, and NFkB p65/p50, whereas EtOH consumption upregulates IKK-α and NFkB p65. **(I-L)** Merged images of NFkB p65 immunofluorescence and DAPI nuclear staining in the OC **(I)**, OC + Mel **(J)**, OC + EtOH **(K)**, and OC + EtOH + Mel groups **(L)**; details of cytosolic/nuclear staining (Alexafluor®488, Bar = 10 μm). EtOH: ethanol; mel: melatonin; IKK-α: inhibitor of NFkB kinase subunit alpha; IkBα: inhibitor of NFkB subunit alpha; NFkB p65: NFkB subunit p65 (RelA); NFkB p50: NFkB subunit p50.

### Mel therapy attenuated TRIF-dependent signaling in OC of EtOH-preferring rats

To investigate the effects of mel on the MyD88-independent signaling pathway, the levels of TRAF6, TRIF, and IRF3 were measured in OC tissues. Interestingly, mel therapy downregulated TRAF6 expression (1.24-fold reduction vs. OC; Table 1, Figure 5A, B, M, N), and no significant difference (P < 0.05) was observed following EtOH intake or the combination of EtOH and mel treatment (Table 1, Figure 5C, D, M, N). Unexpectedly, mel significantly attenuated the MyD88-independent TLR2-/TLR4-mediated signaling pathway by reducing the expression of TRIF and IRF3 in serous papillary OC (1.30- and 1.35-fold reduction vs. OC; Table 1, Figure 5E, F, I, J, M, O, P); thus, mel acted as a repressor of the non-canonical TLR2/TLR4-mediated signaling pathway. Furthermore, mel therapy dramatically reduced the expression of TRIF and IRF3 during EtOH intake (1.55- and 1.28-fold reduction, respectively, vs. OC + EtOH; Figure 5G, H, K, L, M, O, P). As shown in Figure 5Q, mel negatively regulated TRAF6, TRIF, and IRF3 in OC cells and was considered to alter both early and late-phase NFkB translocation and IFN-β production.

**Figure 5:** **Immunohistochemical localization and Western blot analysis of TRAF6, TRIF, and IRF3 in serous papillary ovarian carcinoma.** The immunoreactivity for TRAF6 was moderate in the OC group **(A)** and weak in the OC + Mel group **(B)**. The OC + EtOH **(C)** and OC + EtOH + Mel groups **(D)** displayed weak immunostaining for TRAF6 (arrow). The immunoreactivity for TRIF was enhanced in the epithelium of the OC **(E)** and OC + EtOH groups **(G)**, but mel therapy resulted in weak reaction for TRIF in the OC + Mel **(F)** and OC + EtOH + Mel groups **(H)**. Strong immunoreactivity for IRF3 was observed in the animals from the OC **(I)** and OC + EtOH groups **(K)**, in contrast to the moderate to high reactions in the surface epithelium of the OC + Mel **(J)** and OC + EtOH + Mel groups **(L)** (arrow). Bar = 20 μm. Negative controls were used. **(M)** Representative TRAF6, TRIF, and IRF3 expression profiles in extracts (70 μg protein) pooled from 10 samples/group (upper panel). **(N–P)** Extracts obtained from individual rats were used for densitometric analysis of the TRAF6, TRIF, and IRF3 levels following normalization to a loading control (β-actin). All results are expressed as the means ± SD (n = 10 animals/group). ^a^P < 0.05 vs. OC; ^c^P < 0.05 vs. OC + EtOH. **(Q)** Schematic representation of TLR signaling. MyD88 acts as an essential TIR domain-containing adaptor for the induction of inflammatory cytokines in all TLR subtypes (canonical pathway). In the TLR4-mediated signaling pathway, the TIR domain-containing adaptor TRIF stimulates a MyD88-independent pathway (non-canonical pathway). This signal leads to the activation of IRF3 via TBK1 and IKKƐ/IKKi, facilitating the nuclear translocation of IRF3, which activates the expression of inflammatory factor-related target genes (e.g., IFN-β). Treatment with mel induces the downregulation of TRAF6, TRIF, and IRF3. mel: melatonin; TRAF6: tumor necrosis factor receptor-associated factor 6; TRIF: TIR domain-containing adaptor; TBK-1: TANK-binding kinase 1; IRF3: interferon regulatory factor 3; IFN-β: interferon β.

### The IFN-β, TNF-α, and IL-6 levels were reduced after Mel therapy but not in the presence of EtOH

The concentrations of IFN-β, TNF-α, and IL-6 in the OC group were 100.2 ± 12.0 pg/mL, 121.7 ± 11.8 pg/mL and 147.3 ± 16.2 pg/mL, respectively. Treatment with mel significantly attenuated the increased levels of these proinflammatory cytokines in OC tissue (37.8%, 43.2%, and 44.7% of Group OC, respectively; P < 0.01) (Figure 6A-C). In addition, the IL-8 levels were unchanged for all treatments (Figure 6D). Finally, EtOH consumption in association with OC was unable to alter the levels of these inflammatory cytokines (P > 0.05, Figure 6A-D).

**Figure 6:** **ELISA assays of the IFN-β (A), TNF-α (B), IL-6 (C), and IL-8(D) levels.** Supernatants of ovarian samples (n = 20/group) displaying papillary carcinoma were assessed 60 days after the final dose of mel. ^a^P < 0.01 vs. OC. IFN-β: interferon-β; TNF-α: tumor necrosis factor alpha; IL-6: interleukin-6; IL-8: interleukin-8. All results are expressed as the means ± SD. Two-way ANOVA followed by Tukey test was performed.

## Discussion

We recently demonstrated that long-term mel therapy efficiently reduced the OC size and the incidence of adenocarcinoma in ethanol-preferring animals [12]. Although EtOH consumption has been assumed to inhibit plasma mel levels [26], our data showed that both mel-treated groups maintained their physiological levels at night, even in the presence of EtOH. Importantly, the present study revealed that mel negatively regulates the TLR4-mediated, but not TLR2-mediated signaling pathway in OC of ethanol preferring-rats. In addition, the TRIF signaling pathway was downregulated by mel therapy.

Specifically in OC, a variety of TLRs (including TLR2, TLR3, TLR4, and TLR5) are highly expressed in neoplastic ovarian epithelial cells, indicating poor prognosis [31]. In OC cells, TLR4 has been shown to perform a protumor function and to hamper the efficacy of cancer therapies (e.g., paclitaxel) [3]; conversely, mel significantly reduces TLR4 expression in this rat OC model. Although studies of the role of mel in the anti-tumoral suppression of TLR4/NFkB are scarce, *in vitro* data showed that mel promotes the inhibition of TLR4-mediated inflammatory genes via MyD88-dependent signaling pathway [32], and that mel acts as a TLR4/MyD88 antagonist [33]. Due to its anti-inflammatory properties, mel may be considered as an additional therapy for certain tumors. Interestingly, our results indicated for the first time that mel upregulated TLR2 and that the combination of mel with EtOH caused downregulation of TLR2. These results demonstrate that distinct from its effect on other tissues and under other conditions [11,34], EtOH alone reduces the expression of TLR2 in OC cells. Future studies exploring the effect of mel on genetic TLR2 and TLR4 knockout mice are required to further understand the molecular mechanism(s) by which mel regulates inflammation in OC. The activation of the MyD88 signaling pathway induces tumor cell survival, proliferation, and chemoresistance [3,5,6]. Many studies have reported the ability of mel to modulate the MyD88-dependent signaling pathway [25,32]. MyD88 is a critical adaptor that is directly involved in the TLR4-mediated expression of inflammatory genes [35]. The present study showed that the level of MyD88 was significantly reduced following mel therapy in OC. These results are in agreement with others that showed that mel effectively suppressed the elevation of MyD88 expression in several disorders associated with inflammatory responses [25,32,36]. Conversely, EtOH intake is associated with increased expression of MyD88, mainly in the liver of females exposed to higher doses of EtOH (6 g EtOH/kg b.w.) [37]. Although MyD88 expression appears to be unaffected by EtOH intake, mel therapy significantly inhibited the MyD88-dependent signaling pathway in experimental OC.

NFkB plays a critical role in the TLR4-mediated signaling pathway in tumor cells. Under unstimulated conditions, NFkB is retained in the cytoplasm by binding to IkB. After phosphorylation by IKK, IkB is degraded via the proteasome, and the NFkB subunits p65 and p50 translocate to the nucleus [38]. According to an earlier report involving serous papillary OC, the mechanisms underlying long-term survival and chemotherapy resistance are directly associated with NFkB signaling [39]. The present study showed that mel significantly reduced the expression of IKK-α, IkBα, and NFkB p50/p65 in OC cells. Furthermore, the NFkB subunit p65 was reduced in cytosolic and nuclear extracts, demonstrating that mel may act on mechanisms regulating gene expression and nuclear translocation of NFkB p65. Most of the effects of NFkB activation on tumor cells have been linked to the upregulation of antiapoptotic protein expression, cell proliferation, and proinflammatory cytokine production [5,40], which may enable these cells to progress and metastasize. Thus, we propose that the inhibitory effect of mel on the TLR4-mediated signaling pathway might be partially attributed to the repression of NFkB activation in OC.

Despite the lack of any significant macroscopic or molecular effect of EtOH on OC, chronic EtOH intake caused an elevation in the IKK-α and NFkB p65 levels in animals bearing OC without affecting upstream molecules. In these animals, mel therapy induced the downregulation of NFkB p65 expression but exerted no effect on the IKK-α levels. Indeed, EtOH alone exerts immunomodulatory effects and induces alterations in downstream TLR signaling in many target organs, such as the liver, the brain, and the gastric mucosa [41,42]. These alterations include upregulation of specific cytokines and inflammatory mediators by activating IKKs, MAPKs, and NFkB [42]. Furthermore, TLR4 receptors were reported to be involved in the ethanol-mediated inflammatory response because the blockade of TLR4 abolishes the production of inflammatory mediators and cell death. Although acetaldehyde appears to severely alter TLR4 signaling, the underlying mechanisms by which acetaldehyde targets TLR4 are unknown [43]. Based on our data, we suggest that EtOH intake may affect only some molecules downstream of TLR4 in OC cells, such as the high activity of NFkB p65. Furthermore, EtOH intake exerted no influence on the expression of NFkB-regulated pro-inflammatory cytokines.

TRIF, another adaptor molecule of TLRs, is responsible for the regulation of MyD88-independent pathways [44]. TRIF signals the downstream kinases TBK1 and IKK, leading to phosphorylation of IRF3 and the consequent production of IFNs and IFN-inducible genes [45]. In particular, TRIF/IRF3-dependent signaling is thought to be critical in OC [46]. TRIF contains an N-terminal region termed the effector-driving site that recruits TRAF, resulting in the activation of IRF3 and NFkB [46]. The present study showed that TRAF6, TRIF, and IRF3 were markedly increased in OC and that mel therapy inhibited their expression. Recent studies have elucidated the protective effect of mel on the ischemia/reperfusion-injured liver [25] and on lipopolysaccharide (LPS)-stimulated macrophages by reducing TRIF and IRF3 expression [32]. In EtOH-preferring animals bearing OC, the expression of TRIF and IRF3 was similar to that of the OC group, and mel significantly repressed the expression of these factors. It has been assumed that alcoholism induces an inflammatory process at various levels, depending on the amount of EtOH consumed and the specific tissue [47]. This process may include the production of proinflammatory cytokines that are primarily stimulated by the TLR4/TRIF/IRF3-dependent signaling pathway [47]. Specifically in OC cells, mel therapy led to the downregulation of TRIF and IRF3.

The OC microenvironment is characterized by a dramatic increase in immunosuppressive cytokines, such as TNF-α and IL-6 [46]. These cytokines activate other inflammatory molecules that are capable of recruiting macrophages and dendritic cells (DCs) to the tumor site; these cells further contribute to angiogenesis, tumor growth, and metastasis [48]. Moreover, high levels of anti-inflammatory cytokines and related factors (e.g., TGF-β and VEGF) have been found in OC ascites [49]. Interestingly, we showed a significant reduction in IFN-β, TNF-α, and IL-6 expression in OC after mel therapy. By activating T helper (Th)-1 lymphocytes, mel enhances the production of cytokines such as IL-2, IL-6, IL-12, and IFNs [50], demonstrating its beneficial effects on immune cell modulation. In addition, the anti-inflammatory actions of mel are mediated by multiple mechanisms, including a reduction in the levels of pro-inflammatory cytokines and chemokines (IFNs, TNF-α, IL-6, −8, and −12) and an increase in the levels of anti-inflammatory cytokines (IL-10 and IL-1 antagonist). In OC cells, the immunomodulatory properties of mel may aid in inhibiting tumor cell growth and survival.

## Conclusions

In summary, this study emphasizes the cross-talk between the TLR system and mel in ethanol-preferring rats with OC. Although long-term mel therapy exerts no influence on TLR2 signaling, it may modulate the TLR4-signaling pathway in a MyD88- and TRIF-dependent manner, thereby dampening the inflammatory process induced by OC. Although EtOH alone did not promote additional inflammation in the OC microenvironment, mel therapy efficiently reduced the levels of important inflammatory factors (IkBα, NFkB p65, TRIF, and IRF-3) during EtOH intake. These findings suggest a basis for the therapeutic use of melatonin as a possible adjuvant in association with other anti-cancer therapeutic drugs.

### Summary statement

Melatonin therapy attenuates the TLR4 signaling pathway in a MyD88- and TRIF-dependent manner, dampening the inflammatory process induced by OC in a preclinical model of ovarian carcinogenesis. These findings suggest a basis for the therapeutic use of melatonin as an adjuvant.

### Clinical perspectives

- TLR4-mediated signaling is associated with the immune escape of ovarian cancer cells, and inhibition of specific pro-inflammatory cytokines represents a highly important therapeutic strategy.
- Melatonin, an anti-inflammatory and immunomodulatory indoleamine, modulated the TLR4 signaling pathway, ultimately reducing the expression of inflammation-related mediators in these ovarian cancer cells, which serve as a novel and interesting preclinical model of ovarian cancer.
- These findings suggest a basis for the therapeutic use of melatonin as a possible adjuvant in association with other anti-cancer drugs under investigation in ongoing clinical studies.

## Abbreviations

OC: Ovarian cancer
Mel: Melatonin
EtOH: Ethanol
TLR2: Toll-like receptor 2
TLR4: Toll-like receptor 4
MyD88: Myeloid differentiation factor 88
NFkB: Nuclear factor kappa B
NFkB p65: NFkB subunit p65
NFkB p50: NFkB subunit p50
IkBα: Inhibitor of NFkB alpha
IKK-α: IkB kinase alpha
TRAF6: TNF receptor-associated factor 6
TRIF: Toll-like receptor-associated activator of interferon
IRF3: Interferon regulatory factor 3
IFN-β: Interferon β
TNF-α: Tumor necrosis factor alpha
IL-6: Interleukin 6
IL-8: Interleukin 8
